The article "An Epidemiological Study on the Relationship between Drug Control Program and Patient Compliance in Elderly Patients with Hypertension" was retracted in 2023. Reasons: unreliable results or conclusions; lack of ethics approval or compliance; concerns about the data; concerns about the peer review.

# An Epidemiological Study on the Relationship between Drug Control Program and Patient Compliance in Elderly Patients with Hypertension

**DOI:** 10.1155/2022/7942727

**Published:** 2022-07-30

**Authors:** Yuting Pu, Xinye Wang, Bo Min, Zhibo Sun

**Affiliations:** ^1^School of Health Management, Changchun University of Chinese Medicine, Changchun 130000, Jilin, China; ^2^JiLin Province FAW General Hospital, Changchun 130000, Jilin, China

## Abstract

**Objective:**

To explore the relationship between medication control regimen and patient compliance in elderly hypertensive patients.

**Methods:**

A retrospective analysis of 1432 elderly hypertensive patients in our hospital from February 2020 to February 2021 was conducted. The general data of patients, the drug control regimen, the occurrence of drug side effects, and blood pressure control of patients during hospitalization and outpatient follow-up were statistically analyzed.

**Results:**

The first dose rate was higher in patients given a single dose during hospitalization than in patients followed up in outpatient clinics, and the discharge rate was lower than for single doses (*P* < 0.05). Patients had a lower first dose rate and a higher discharge rate for the two drug combinations during hospitalization compared to outpatient follow-up patients, while the first dose rate and discharge rate were significantly lower during hospitalization. Three drugs were administered (*P* < 0.05). A higher incidence of first-dose and discharge medication was observed in patients with four drug coadministration during hospitalization than in patients with outpatient follow-up. The incidence of angiotensin-converting enzyme inhibitors (dry cough) was higher and the incidence of diuretics (hypokalemia) was lower in patients during hospitalization compared with patients at outpatient follow-up (*P* < 0.05). Maximum systolic blood pressure and fluctuations in systolic and diastolic blood pressure were lower in well compliant patients than in poorly compliant patients (*P* < 0.05). First systolic, maximal systolic, first diastolic, maximal diastolic, systolic and diastolic fluctuations were higher in hospitalised patients than in patients with outpatient follow-up, regardless of treatment compliance (*P* < 0.05).

**Conclusion:**

Elderly hypertensive patients with outpatient follow-up had the best discharge medication compliance, patients during hospitalization showed good medication compliance, and patients with outpatient follow-up had poor medication compliance.

## 1. Introduction

Hypertension is extremely common in China, with the number of patients reaching 200 million [1], and is highly predisposed to complications such as heart disease and stroke. In recent years, the number of elderly patients with hypertension has shown an increasing trend. As the elderly age, they begin to show signs of arterial wall sclerosis and reduced vascular compliance and elasticity, which will lead to a decrease in the vascular regulation of blood pressure, resulting in hypertension [2]. In addition, the elderly may experience structural changes in the heart, such as fibrosis of the left ventricular myocardium, thickening of the ventricular wall, and reduced compliance, which may lead to reduced diastolic and systolic function in the elderly with hypertension, resulting in cardiac insufficiency and arrhythmias [3]. In addition, prolonged hypertension can cause hypertension to be exacerbated by reduced renal function [4]. In elderly patients with hypertension, pressure receptor sensitivity is reduced, making the elderly less able to buffer and regulate fluctuations in blood pressure [5]. In addition, vascular sclerosis, reduced compliance, and endothelial abnormalities reduce the ability to regulate intravascular pressure changes [6].

The article "An Epidemiological Study on the Relationship between Drug Control Program and Patient Compliance in Elderly Patients with Hypertension" was retracted in 2023. Reasons: unreliable results or conclusions; lack of ethics approval or compliance; concerns about the data; concerns about the peer review.

The primary goals of hypertension treatment in the elderly are to control blood pressure, protect target organs, and minimise the risk of cardiovascular and cerebrovascular events and death. The main components include lifestyle interventions and pharmacological treatment. Antihypertensive drug therapy includes five major classes of calcium antagonists, angiotensin-converting enzyme inhibitors, beta-blockers, angiotensin receptor blockers, and diuretics [7]. Small to moderate doses of statins can achieve the total and LDL cholesterol targets in most elderly patients [8]. Elderly hypertensive patients with comorbid diabetes mellitus should be better monitored with glucose-lowering drugs [9]. The use of low-dose aspirin in elderly hypertensive patients at high risk of cardiovascular disease may reduce the risk of cardiovascular events, but its use should be carefully assessed after being informed of the risks and risk factors, and bleeding tendencies and adverse effects should be monitored during administration [10]. Previous research has indicated that prevention of further development of the disease entails timely anti-hypertensive drug therapy [11]. However, a common problem with clinical medication use is poor patient adherence. Therefore, this study investigated a medication control regimen for hypertension in older adults and examined the potential relationship between the regimen and patient adherence.

## 2. Materials and Methods

### 2.1. General Information

The clinical data of 1432 cases of elderly hypertensive patients in our hospital (JiLin Province FAW General Hospital) from February 2020 to February 2021 were retrospectively analyzed.

The article "An Epidemiological Study on the Relationship between Drug Control Program and Patient Compliance in Elderly Patients with Hypertension" was retracted in 2023. Reasons: unreliable results or conclusions; lack of ethics approval or compliance; concerns about the data; concerns about the peer review.

Inclusion criteria: (1) Patients were aged 60 years and above; (2) Patients who met the diagnostic criteria for essential hypertension [12]. Exclusion criteria: (1) Patients with malignant tumors; (2) Patients who withdrew midway.

### 2.2. Methods

The medication control regimen and the occurrence of medication side effects were investigated in 1432 elderly patients with hypertension and 914 patients with outpatient follow-up, and the changes in blood pressure levels were observed in patients with both good and poor treatment compliance (Good treatment compliance: patients took the medication as prescribed, without random addition, subtraction or change in medication, were able to tolerate medication side effects and had ideal blood pressure control. Poor treatment compliance: patients increased, subtracted, or changed medication when they were unable to tolerate medication side effects or lacked ideal blood pressure control [13]).

### 2.3. Observational Indicators

(1) General information; (2) drug control regimen; (3) occurrence of drug side effects; and (4) blood pressure control.

### 2.4. Statistical Analyses

SPSS 21.0 was used for data analysis. Count data were expressed as rates and analyzed using the *χ*2 test or rank-sum test. The measurement data were expressed as ($\bar{x}\pm s$) and analyzed using the *t*-test or F-test. *α* = 0.05 was used as a criterion for statistically significant differences in comparisons.

## 3. Results

### 3.1. General Information Analysis

There were 408 females and 1024 males aged 63–83 years, with a mean age of 46.25 ± 7.35 years. The subjects had 1006 cases aged 63 to 73 years and 426 cases aged 74 to 83 years in terms of age distribution; 732 cases between 1 month and 14 years and 700 cases between 15 and 35 years in terms of the duration of hypertension; 510 cases of grade I, 602 cases of grade II, and 320 cases of grade III in terms of hypertension classification; 440 cases with a family history of hypertension; and 992 cases without a family history of hypertension in terms of family history of hypertension. 1176 cases with diagnosis at admission and 256 cases with diagnosis after admission in terms of the time of diagnosis; 436 cases from rural areas and 690 cases from urban areas in terms of residence; 64 cases of illiterate, 690 cases of elementary school, 402 cases of secondary school, and 276 cases of university and above in terms of educational level; 956 cases of smoking, 852 cases of lipid metabolism disorders, 558 cases of diabetes mellitus, 136 cases of left ventricular hypertrophy, 108 cases of renal impairment, and 82 cases of transient ischemic attack or stroke in terms of risk factors; and 914 cases with outpatient follow-up and 518 cases without in terms of outpatient follow-up. The elderly hypertensive patients were mainly men aged 63–73 years, most of whom had no family history of hypertension, with diagnosis after admission, urban residence, elementary school education, and outpatient follow-up, and the main risk factors were smoking, lipid metabolism disorders, and diabetes mellitus as shown in Table 1.

The article "An Epidemiological Study on the Relationship between Drug Control Program and Patient Compliance in Elderly Patients with Hypertension" was retracted in 2023. Reasons: unreliable results or conclusions; lack of ethics approval or compliance; concerns about the data; concerns about the peer review.

### 3.2. Comparison of Drug Control Regimens

Patients during hospitalization had a higher rate of first dosing and a lower rate of discharge medication than outpatient follow-up patients in single drug administration (*P* < 0.05). In contrast to the outpatient follow-up patients, patients during hospitalization had a lower rate of first dose and a higher rate of discharge medication in the coadministration of two drugs, and significantly lower rates of first dose and discharge medication in the coadministration of three drugs (*P* < 0.05). A high rate of first dose and discharge medication was observed in the patients during hospitalization in the coadministration of four drugs than the outpatient follow-up patients (*P* < 0.05). See Tables2 and 3.

### 3.3. Comparison of the Incidence of Drug Side Effects

Patients during hospitalization showed a higher incidence of angiotensin-converting enzyme inhibitors (dry cough) and a lower incidence of diuretics (hypokalemia) than outpatient follow-up patients (*P* < 0.05). The difference between the incidence of Β blockers (bradycardia) and calcium antagonists (swelling/flushing/tachycardia) was not significant in patients (*P* > 0.05) as shown in Table 4.

### 3.4. Comparison of Blood Pressure Control

The maximum systolic blood pressure and the range of systolic and diastolic fluctuations were lower in patients with good compliance than in patients with poor compliance (*P* < 0.05), but no significant differences were found in the first systolic blood pressure, minimum systolic blood pressure, first diastolic blood pressure, maximum diastolic blood pressure, minimum diastolic blood pressure, and final blood pressure between them (*P* > 0.05). The first systolic, maximum systolic, first diastolic, maximum diastolic, and systolic and diastolic ranges of fluctuation were higher in patients during hospitalization than in outpatient follow-up patients regardless of treatment compliance (*P* < 0.05), but the differences in the minimum systolic blood pressure, minimum diastolic blood pressure, and final blood pressure were not significant between them (*P* > 0.05) as shown in Tables 5–7.

The article "An Epidemiological Study on the Relationship between Drug Control Program and Patient Compliance in Elderly Patients with Hypertension" was retracted in 2023. Reasons: unreliable results or conclusions; lack of ethics approval or compliance; concerns about the data; concerns about the peer review.

## 4. Discussion

The results of this study showed that elderly patients with hypertension were predominantly male, aged between 63 and 73 years, most without a family history of hypertension, diagnosed after hospital admission, urban residence, primary school education, outpatient follow-up, and the main risk for factors including smoking, lipid metabolism disorders, and diabetes mellitus. In general, the first inpatient dosing started with a single dose, which was adjusted in real time during the hospital stay according to the patient's blood pressure control. Once blood pressure is stable, patients are discharged from hospital with a combination of 2 antihypertensive drugs, followed by a single dose, and finally a combination of 3 or more antihypertensive drugs. The outpatient follow-up started with mainly a combination of 2 anti-hypertensive drugs, and at the last visit, single administration was mainly given, followed by a combination treatment of 2 anti-hypertensive drugs [14, 15]. Patients during hospitalization had a higher rate of first dosing and a lower rate of discharge medication than outpatient follow-up patients in single drug administration (*P* < 0.05). In contrast to the outpatient follow-up patients, patients during hospitalization had a lower rate of first dose and a higher rate of discharge medication in the coadministration of two drugs, and significantly lower rates of first dose and discharge medication in the coadministration of three drugs (*P* < 0.05). The first dose and discharge dosing rates were higher in patients on the combination of the four drugs during hospitalization than in patients followed up in outpatient clinics, indicating that elderly hypertensive patients followed up in outpatient clinics had the best adherence to their medication at discharge.

It has been reported [16–19] that outpatient follow-up patients experienced fewer drug side effects with angiotensin-converting enzyme inhibitors and more drug side effects with diuretics than patients during hospitalization. Results of this study demonstrated that patients during hospitalization showed a higher incidence of angiotensin-converting enzyme inhibitors (dry cough) and a lower incidence of diuretics (hypokalemia) than outpatient follow-up patients (*P* < 0.05), which is consistent with previous research. Previous studies [20–22] have shown that compliance with antihypertensive medication for hypertension ranges from 50% to 84%. Poor adherence to treatment during hospitalization was mainly seen in secondary school students and urban patients due to medication side effects and poor blood pressure control, whereas poor adherence to discharge medication was mainly seen in primary school and rural patients due to subjective factors, financial factors, medication side effects, and lack of satisfactory blood pressure control. Poor treatment compliance during outpatient follow-up was mostly recorded in middle and elementary school-educated and rural patients due to subjective factors, economic factors, physician factors, medication side effects, and lack of ideal blood pressure control [23–25]. Herein, the maximum systolic blood pressure and the range of systolic and diastolic fluctuations were lower in patients with good compliance than in patients with poor compliance (*P* < 0.05). Regardless of treatment compliance, inpatients had higher fluctuations in first systolic, maximal systolic, first diastolic, maximal diastolic, systolic and diastolic blood pressures than patients followed up in outpatient clinics (*P* < 0.05), which was attributed to poor intermittent treatment compliance with anti-hypertensive medication and frequent changes in medication type, resulting in sustained poor blood pressure control. In addition, given the significant blood pressure fluctuations in hypertensive patients, treatment irregularities strongly predispose to damage of hypertensive target organs [26–29].

The article "An Epidemiological Study on the Relationship between Drug Control Program and Patient Compliance in Elderly Patients with Hypertension" was retracted in 2023. Reasons: unreliable results or conclusions; lack of ethics approval or compliance; concerns about the data; concerns about the peer review.

Compared with Western medicine, many elderly people prefer and trust Chinese medicine treatment methods [30]. Hypertension belongs to the category of vertigo in TCM [31]. The general drugs for the treatment of senile hypertension are as follows: (1) Chaihu-Shugan-San (CHSGS) is a commonly used traditional Chinese medicine for the treatment of senile hypertension. After taking the medicine, it can not only lower blood pressure but also relieve the severe headache caused by high blood pressure [32]. (2) Qiju Dihuang Decoction has the functions of clearing liver and cooling blood, reducing fire and diuresis, and clearing heat, inducing heat and reducing heat pressure effect. After taking the medicine, it can quickly relieve the problem of high blood pressure and treat constipation, dizziness, and other adverse conditions [33]; (3) Erxian Decoction can also be used to treat hypertension in the elderly. The function of conditioning Chong and Ren to lower blood pressure is quite significant [34]. Hypertensive patients can use some acupuncture and moxibustion as adjuvant therapy at ordinary times. The acupuncture and moxibustion treatment can choose different acupuncture points or acupuncture methods for different constitutions of their own patients [35]. It is generally a benign stimulation, which can clear the meridians and nourish the liver and kidney, which can make the patient's qi and blood unobstructed. Generally, the blood pressure will gradually decrease, and there are no side effects [36]. The clinical use of traditional Chinese medicine to treat elderly patients or the use of integrated traditional Chinese and Western medicine may improve the compliance of elderly patients with medication.

The article "An Epidemiological Study on the Relationship between Drug Control Program and Patient Compliance in Elderly Patients with Hypertension" was retracted in 2023. Reasons: unreliable results or conclusions; lack of ethics approval or compliance; concerns about the data; concerns about the peer review.

## 5. Conclusion

In conclusion, elderly hypertensive patients with outpatient follow-up had the best discharge medication compliance, patients during hospitalization showed good medication compliance, and patients with outpatient follow-up had poor medication compliance.

## Figures and Tables

**Table 1:** Analysis of general information.

Index	Categories	Distribution	Item	Categories	Distribution
Age (years)		46.25 ± 7.35	Place of residence	Rural	436 (30.4)
Gender	Female	408 (28.5)		Urban	996 (69.6)
	Male	1024 (71.5)	Education level	Illiterate	64 (4.5)

Age distribution	63∼73 years old	1006 (70.3)		Elementary	690 (48.2)
	74∼83 years old	426 (29.8)		Secondary school	402 (28.1)

Duration of hypertension	1 month∼14 years	732 (51.1)		University and above	276 (19.3)
	15∼35 years	700 (48.9)	Outpatient follow-up	Yes	914 (63.8)

Hypertension classification	Grade I	510 (35.6)		No	518 (36.2)
	Grade II	602 (42.0)	Risk factors	Smoking	956 (66.8)
	Class III	320 (22.3)		Lipid metabolism disorder	852 (59.5)

Family history of hypertension	Yes	440 (30.7)		Diabetes mellitus	558 (39.0)
	No	992 (69.3)		Left ventricular hypertrophy	136 (9.5)

Diagnosis time	Upon admission	1176 (82.1)		Renal impairment	108 (7.5)
	After admission	256 (17.9)		Transient ischemic attack or stroke	82 (5.7)
				Peripheral vascular lesions	58 (4.1)

**Table 2:** Comparison of single drug administration in drug control regimens (*n* (%)).

Groups	*n*	Time	Angiotensin-converting enzyme inhibitors	Β-blockers	Calcium antagonists	Diuretics	Total
During hospitalization	1432	First dosing	280 (19.6)	134 (9.4)	242 (16.9)	48 (3.4)	704 (49.2)
		Discharge medication	242 (16.9)	144 (10.1)	216 (15.1)	40 (2.8)	642 (44.8)

Outpatient follow up	914	First dosing	102 (11.2)	56 (6.1)	100 (10.9)	42 (4.6)	300 (32.8)
		Discharge medication	152 (16.6)	86 (9.4)	154 (16.8)	72 (7.9)	460 (50.3)

**Table 3:** Comparison of coadministration in drug control regimens (*n* (%)).

Groups	*n*	Time	Coadministration of two drugs	Coadministration of three drugs	Coadministration of four drugs
During hospitalization	1432	First dosing	502 (35.1)	198 (13.8)	28 (2.0)
		Discharge medication	520 (36.3)	230 (16.1)	40 (2.8)

Outpatient follow up	914	First dosing	378 (41.4)	228 (24.9)	8 (0.9)
		Discharge medication	216 (23.6)	232 (25.4)	6 (0.7)

**Table 4:** Comparison of the incidence of drug side effects ($\bar{x}\pm s$).

Groups	*n*	Angiotensin-converting enzyme inhibitors (dry cough)		Β*B* blockers (bradycardia)		Calcium antagonists (swelling/flushing/tachycardia)		Diuretics (hypokalemia)	
During hospitalization	1432	712	92 (12.9)	304	44 (15.2)	732	70 (9.6)	246	24 (9.8)
Outpatient follow up	914	490	42 (8.6)	196	24 (14.3)	472	48 (10.2)	204	60 (29.4)

The article "An Epidemiological Study on the Relationship between Drug Control Program and Patient Compliance in Elderly Patients with Hypertension" was retracted in 2023. Reasons: unreliable results or conclusions; lack of ethics approval or compliance; concerns about the data; concerns about the peer review.

**Table 5:** Comparison of blood pressure control (mmHg, $\bar{x}\pm s$).

Groups	*n*	Treatment compliance	First systolic blood pressure	Maximum systolic blood pressure	Minimum systolic blood pressure
During hospitalization	1432	Good	150.4 ± 18.6	150.5 ± 10.8	125.0 ± 16.8
		Poor	152.0 ± 17.8	167.3 ± 14.1	124.5 ± 14.1

Outpatient follow-up	914	Good	123.1 ± 12.0	130.0 ± 7.1	122.2 ± 14.8
		Poor	124.3 ± 11.8	138.1 ± 13.4	124.4 ± 8.1

**Table 6:** Comparison of blood pressure control (mmHg, $\bar{x}\pm s$).

Groups	*n*	Treatment compliance	First diastolic blood pressure	Maximum diastolic blood pressure	Minimum diastolic blood pressure
During hospitalization	1432	Good	95.5 ± 15.5	95.8 ± 9.1	77.4 ± 10.2
		Poor	96.6 ± 12.8	97.4 ± 9.8	72.7 ± 8.8

Outpatient follow-up	914	Good	74.1 ± 10.1	80.1 ± 8.0	71.7 ± 7.0
		Poor	72.2 ± 10.8	84.4 ± 8.8	71.8 ± 8.7

**Table 7:** Comparison of blood pressure control (mmHg, $\bar{x}\pm s$).

Groups	*n*	Treatment compliance	Range of fluctuation		Final blood pressure	
			systolic blood pressure	diastolic blood pressure	systolic blood pressure	diastolic blood pressure
During hospitalization	1432	Good	25.4 ± 4.4	18.3 ± 1.4	132.0 ± 9.4	79.0 ± 10.0
		Poor	42.7 ± 5.7	24.6 ± 3.4	133.1 ± 9.1	78.0 ± 9.1

Outpatient follow-up	914	Good	7.8 ± 1.0	8.3 ± 1.0	125.0 ± 7.7	73.8 ± 6.4
		Poor	13.6 ± 4.5	16.5 ± 2.8	126.8 ± 8.0	75.8 ± 8.0

## Data Availability

No data were used to support this study.
